The article "Differential SELEX in Human Glioma Cell Lines" was retracted in 2020. Reasons: manipulated images; duplicated images; original data or images not available; concerns about the results or conclusions.

# Differential SELEX in Human Glioma Cell Lines

**DOI:** 10.1371/journal.pone.0007971

**Published:** 2009-11-24

**Authors:** Laura Cerchia, Carla Lucia Esposito, Andreas H. Jacobs, Bertrand Tavitian, Vittorio de Franciscis

**Affiliations:** 1 Istituto per l'Endocrinologia e l'Oncologia Sperimentale del CNR “G. Salvatore”, Naples, Italy; 2 Dipartimento di Biologia e Patologia Cellulare e Molecolare, Università di Napoli “Federico II”, Naples, Italy; 3 European Institute of Molecular Imaging (EIMI), University of Muenster, Muenster, Germany; 4 Laboratory for Gene Therapy and Molecular Imaging, Max Planck Institute for Neurological Research, Cologne, Germany; 5 CEA/DSV/DRM Service Hospitalier Frederic, Joliot, INSERM ERM 103, Orsay, France; University of Hong Kong, Hong Kong

## Abstract

The hope of success of therapeutic interventions largely relies on the possibility to distinguish between even close tumor types with high accuracy. Indeed, in the last ten years a major challenge to predict the responsiveness to a given therapeutic plan has been the identification of tumor specific signatures, with the aim to reduce the frequency of unwanted side effects on oncologic patients not responding to therapy. Here, we developed an *in vitro* evolution-based approach, named differential whole cell SELEX, to generate a panel of high affinity nucleic acid ligands for cell surface epitopes. The ligands, named aptamers, were obtained through the iterative evolution of a random pool of sequences using as target human U87MG glioma cells. The selection was designed so as to distinguish U87MG from the less malignant cell line T98G. We isolated molecules that generate unique binding patterns sufficient to unequivocally identify any of the tested human glioma cell lines analyzed and to distinguish high from low or non-tumorigenic cell lines. Five of such aptamers act as inhibitors of specific intracellular pathways thus indicating that the putative target might be important surface signaling molecules. Differential whole cell SELEX reveals an exciting strategy widely applicable to cancer cells that permits generation of highly specific ligands for cancer biomarkers.

## Introduction

A major challenge in oncology aims at the characterization of the heterogeneity of disease by defining more reliable diagnostic/prognostic factors and at developing effective anticancer therapeutics selectively targeting tumor cells. Indeed, cancer is a complex disease characterized by the accumulation of several and often unknown molecular alterations that cause genetic instability, cell proliferation, and acquisition of an increasingly invasive phenotype resistant to therapeutic treatments. In turn the heterogeneity of malignant cells combined to the variability of the patient's genetic background create different cancer phenotypes with distinct clinical outcomes. By reducing the degree of uncertainty on the clinical status of individual patients, the simultaneous analysis of multiple biomarkers improves the possibility to distinguish between two even close tumor types and predict distinct therapeutic responses.

Aptamers are small and highly structured single-stranded oligonucleotides that bind at high affinity (within the low nanomolar range) to a target molecule by providing a limited number of specific contact points imbedded in a larger, defined three-dimensional structure [1], [2], [3], [4], [5].

Aptamers are isolated by the Systematic Evolution of Ligands by EXponential enrichment (SELEX) technology and since from their first description in 1990 [1], [6], aptamers soon became a valuable research tool and show great application prospected in fundamental research, drug selection and clinical diagnosis and therapy. At present, aptamers against many kinds of proteins have come into clinical test phase [7], [8], [9].

Recently, nucleic acid aptamers have been selected against whole living cells, with the advantage of a direct selection of ligands without prior knowledge of the target molecules, notably by using as target red blood cells [10], leukemia cells [11] small lung cancer cells [12] and rat brain tumor microvessels [13]. Nonetheless, the use of complex cells as targets has been shown to enable the identification of aptamers that bind large cell surface-specific markers, in their native conformation.

Indeed, by applying SELEX technology against whole-living cells in culture, for the first time we succeeded in demonstrating that even by using complex targets as intact cells, it is possible to obtain aptamers against even rare antigens if specifically expressed on the target cell [14]. We adopted this strategy to generate nuclease resistant RNA-aptamers specific for PC12 cells expressing the human receptor tyrosine kinase, Ret and selected aptamers that bind specifically to Ret and inhibit its downstream signaling effects [14].

Herein, we have developed a whole-cell SELEX protocol with the aim to generate aptamers able to discriminate within the same tumor between two strictly related phenotypes. We used glioblastoma cell lines as model system because of the complex cellular heterogeneity of malignant gliomas and the need to find new diagnostic and therapeutic modalities for these tumors. By using a counterselection/selection approach, specifically designed to enrich for aptamers against cell surface tumor-specific targets, we have generated a panel of RNA-aptamers able to bind at high affinity to malignant U87MG cells. They do not bind the non tumorigenic T98G nor other non-related cancer cell types, but bind to glioma cell lines characterized by different malignant phenotypes at different extents. Furthermore, functional analysis revealed that some of the aptamers inhibit specific intracellular signaling pathways.

Our results indicate the differential whole-cell SELEX strategy as a promising strategy to develop specific molecular probes for early diagnosis and prediction of aggressiveness and therapeutic response that is generally applicable to different strictly related cell types.

## Results

### Enrichment of Selection for a Complex Target

In order to isolate cell specific ligands for a given tumor cell phenotype we decided to keep as model system stable human glioma cell lines. Even though using stable cell lines has the drawback of skipping epitopes that might be important for the *in vivo* cell growth, it has the obvious advantage to handle a cell population under well controlled growth conditions that remain stable all along the SELEX procedure. We used as target for the selection steps the malignant human U87MG glioma cell line and for the counterselection steps less malignant human T98G glioma cells. These two cell lines differ for the potential to form tumors in nude mice, U87MG being highly tumorigenic while the T98G are poorly tumorigenic. On the other hand, these cell lines share same cellular pathways altered, both harboring p14^arf^/p16 deletion and phosphatase and tensin homolog (PTEN) mutation. Major differences found between the two cell lines are the levels of ErbB2 and of phosphorylated extracellular signal-regulated protein kinase (ERK), that are higher in U87MG than in T98G, while phosphorylated Akt and neural cell adhesion molecule (NCAM) levels were similar (data not shown). The relative levels of these four molecules were monitored at each cycle of the SELEX procedure to verify and standardize the growth conditions of the cells.

A library of 2'Fluoro Pyrimidines (2'F-Py), nuclease-resistant RNAs was utilized for differential SELEX against intact cells (Fig. 1). At each round the selection step on U87MG cells was preceded by one or two counterselection steps against T98G cells. During the selection process, we progressively increased the selective pressure by changing both incubation and washing conditions. During rounds 13 and 14, restriction fragment length polymorphism analysis (RFLP) profiles remain unchanged, suggesting that the population had stopped to evolve under the selection pressure (data not shown). Indeed, as assessed by comparing the *in vitro* binding efficiency on the two cell lines and to the naïve starting pool (not shown), after 14 rounds of selection, the pool, named G14, was enriched for aptamers that preferentially bind to U87MG cells.

**Figure 1:** Selection of U87MG cell-specific aptamers. A pool of 2'F-Py RNAs was incubated with poorly tumorigenic T98G cells (Counterselection). Unbound sequences in the supernatant were recovered and incubated with tumorigenic U87MG cells for the selection step (Selection). Unbound sequences were discarded by washings and bound sequences were recovered by total RNA extraction. Sequences enriched by the selection step were amplified by RT-PCR and in vitro transcription before a new cycle of selection.

### Distribution of Individual Sequences

In order to isolate individual aptamers that may distinguish the more malignant U87MG phenotype, a panel of 71 sequences was cloned from the pool G14, and aptamers grouped in families based on their primary sequence similarity (Fig. 2). We identified ten families of highly related aptamers that together cover more than 46% (33 aptamers) of all individual sequences obtained from the selection; one single individual sequence dominated the selection and constituted 8% of all the clones; five other sequences represented together more than 15% of the clones. The remaining 38 sequences were poorly related to each other (Fig. 2).

**Figure 2:** Analysis of individual sequences similarity. Dendogram (obtained by using DNASIS software version 2.1) for visual classification of similarity among 71 individual sequences cloned after 14 rounds of selection. Aptamers are grouped in 10 families of sequences found more than once (labeled with the asterisk) or that share sequence similarity (boxed).

We thus screened for those aptamers that efficiently target the U87MG cells. To this aim a panel of 21 individual aptamers, including at least one member for each family, was analysed for binding at the concentration of 500 nM. At that concentration, 8 aptamers display up to five-fold increase of binding to U87MG cells with respect to the starting pool, while the remaining 13 aptamers show no specific binding to U87MG (not shown). Using the starting pool as control of background, the binding affinity of individual aptamers to U87MG cells and T98G cells was then determined. As shown in Table 1, all 8 sequences (GL17, GL56, GL62, GL36, GL35, GL43 GL44 and GL21) bind at high affinity (with Kd ranging between 33 nM and 700 nM) to the U87MG cells and have no or low affinity for T98G (not shown). Michaelis-Menten binding curves of three aptamers are shown in Fig. 3*A*. Given the good specificity and high affinity for the U87MG cells we restricted our further analysis of biochemical and biological properties to these 8 sequences.

**Figure 3:** Dissociation constants of GL35, GL36, GL21 and GL44-43 short aptamers. (*A*) Binding curve of GL35, GL36 and GL21 aptamers on U87MG. Lineweaver-Burk analysis (inset) was used for the evaluation of the binding constant (see Materials and Methods). (*B*) Secondary structure of a shortened sequence consisting of residues 1–39 of GL44 or GL43 aptamers (GL44-43 short). predicted by using MFOLD software version 3.1 (available at http://www.bioinfo.rpi.edu/applications/mfold/). (*C*) Binding curve of the GL44-43 short aptamer on U87MG cells.

**Table 1:** Sequence of indicated aptamers; for simplicity fixed-primer sequences at 5′ and 3′ are not shown.

	Binding affinity of individual aptamers to U87MG cells	
Name	Sequence	Kd (nM)
**GL17**	CCGUUGUUCUACAUGUCACUCAUCACGCGAGUCUUUUGUCUAA	102±12
**GL21**	GCCUCUCAACGAUUAAUGUUUCGUUAACAUGAUCAAUCGCCUCAA	221±25
**GL62**	UUCACACACUCAAUUGAACGGUGAUUCAAGUUAUUAGCAGCCUCA	710±40
**GL43**	ACGUUACUCUUGCAACAC–AAACUUUAAUAGCCUCUUAUAGUUC	44±4
**GL44**	ACGUUACUCUUGCAACACCCAAACUUUAAUAGCCUCUUAUAGUUC	38±3
**GL56**	UGAUUUUGCAGCACUUCUUGUUAUCUUAACGAACUGUUGAUGA	63±9
**GL36**	UACCAAACGCGCAAUUUUCAUCUUGUAAUAACCAAAUGCCUCUGA	190±20
**GL35**	UACCAAACGCGCGGUUUUCGUCUCGUAAUAACCAAAUGCCUCUGA	44±7

Residues that differ among the sequences in the couple (GL43 and GL44) or (GL36 and GL35) are in bold.

Michaelis-Menten binding curves to estimate Kd (nM) were performed as described in Materials and Methods; standard deviation values were determined from at least four independent experiments.

### Comparison of Individual Sequences

Four of the eight aptamers considered (GL21, GL17, GL56 and GL62) have unrelated primary sequences and predicted 2D folded structures. Two (GL44 and GL43) differ for the presence of two cytosines (cyt42 and cyt43) that are only present in GL44 whose presence however does not alter the affinity for the target cells (see Table 1). Comparing the predicted secondary structures defined a conserved stem-loop (residues 1–39) presents with an identical sequence in both aptamers (Fig. 3*B*). Consistently the shortened sequence, constituted of the first shared 39 residues (herein named GL44-43 short), is sufficient to bind to the U87MG cells displaying a Kd of 30 nM (Fig. 3*C*) and discriminate them from T98G cells (not shown). The opposite situation was found in another couple of aptamers (GL35 and GL36) that even if poorly differ in their primary structures, have binding affinities that differ of around 4 times (Table 1).

### Binding Specificity

The identification of a small set of aptamers that may distinguish the U87MG cells from the T98G cells raises the obvious question of whether these aptamers may bind as well other cell types. To this aim we determined the relative binding potential of each aptamer to several cell lines. We first determined the cell type specificity by measuring at the same concentration of 50 nM the binding of each aptamer on a panel of unrelated cell lines. We found that any of the eight aptamers did not bind to other human cancer cell types analyzed including neuroblastoma (SK-N-BE and SH-SY5Y), lung (H460 and Calu1) and breast (MCF7 and SKBR3) cancer cells nor to murine fibroblast NIH3T3 cells, as assessed by comparison with the unspecific binding of the starting pool, G0 data not shown). On the other hand, even if at different extents they bind to various glioma cell lines (U251MG, TB10, LN-18 and LN-229) and a U87MG derivative, U87MGΔEGFR, but not the T98G cells used for counterselection. These cell lines are characterized by different tumor type derivation and malignant phenotypes and have different genetic backgrounds. As shown in Fig. 4A, at that concentration each aptamer has a distinct pattern of binding on different glioma cell lines (see Legend). At these experimental conditions, all aptamers have good binding with the highly tumorigenic cell lines (U87MG, LN-229, U87MGΔEGFR and TB10), the aptamers GL56 binds to all cell lines except to the non tumorigenic T98G, and GL17 binds only the four highly tumorigenic cell lines. Thus the pattern of binding of five of these aptamers (for example, GL44, GL17, GL56, GL36 and GL35) is sufficient to distinguish two cell lines. Further we confirmed that aptamers can distinguish tumorigenic from non tumorigenic glioma cells by determining binding of four of them (GL21, GL35, GL36 and GL44-43 short) to highly tumorigenic cell lines (U87MG, Gli36, and Gli36ΔEGFR) as compared to two cell lines (A172 and T98G) that are unable to form tumors in nude mice (Fig. 4*B*). Furthermore, the eight aptamers bind also to primary cell cultures of malignant glioblastomas and discriminate them from a not-related meningeoma cell line, thus excluding the recognition of possible unwanted epitopes enriched upon immortalization of a stabilized cell line (Fig. 4*C*). For each aptamer the differences observed in the extent of binding likely reflect the relative concentrations of the same target molecules in the different cell lines.

**Figure 4:** Binding analyses of the best sequences to glioma cell lines. The indicated aptamers or the starting pool (G0) were 5′- [^32^P]-labeled and incubated in the same condition at 50 nM with the indicated stable glioma cell lines (*A and B*) or primary cultures of malignant glioma cells (*C*). The results are expressed relative to the background binding detected with the starting pool. In (*A*) and (*B*) the tumorigenic potential in nude mice is indicated on the basis of the time of appearance of tumor and the tumor growth rate as previously reported [15], [23], [31], [32]: high tumorigenicity is indicated as “++”; middle tumorigenicity is indicated as “+” and no tumorigenicity is indicated as “-”. In (A), the binding capacity of the aptamers to the cells is reported: high binding (more than four-fold) is indicated as “++”, middle binding (between two and four-fold) is indicated as “+” and no binding (less than two-fold) is indicated as “-”.

### Biological Activities of Aptamers

As previously demonstrated for the anti Ret receptor tyrosine kinase D4 aptamer, high affinity aptamer binding to an extracellular receptor may inhibit activity of key downstream transducing molecules, such as ERK family members. Therefore, we first determined whether treating the U87MG cells with any of these aptamers may affect the phosphorylation of either Akt and ERK 1/2.

Treating cells with five aptamers (GL36, GL35, GL44, GL43 and GL21) at 200 nM inhibited ERK phosphorylation of at least two-fold, as compared to the control starting pool and to the other aptamers (GL17, GL56, GL62) (not shown). On the other hand, no aptamer had any relevant effect on the phosphorylation of Akt and of the 3-Phosphoinositide-dependent protein kinase-1 (PDK1) (not shown), most likely because the U87MG harbor a mutated inactive phosphatase and tensin homolog (PTEN), a phosphatase that dephosphorylates the phosphatidylinositol (3,4,5)-trisphosphate, thus resulting in inhibition of the Akt signaling pathway [15].

To further confirm the biological activity of GL36, GL35, GL44, GL43 and GL21, we determined the extent of inhibition of expression of the cell cycle-related protein, cyclin D1 and of phosphorylation of ERK 1/2 upon treatment of U87MG cells with aptamers for increasing time periods.

The cyclin D1 proto-oncogene is an important regulator of G1 to S-phase transition, causing downregulation of protein levels through its protein expression and through phosphorylation-dependent degradation, and causing inhibition of cell cycle progression by inducing a G1 arrest [16], [17]. We thus performed time-course experiments with the five inhibitor aptamers looking at its protein expression and phosphorylation levels. As shown in Fig. 5*A*, treatment with cognate aptamers either GL36 and GL35, or GL44 and GL43, inhibits at similar extents basal cyclin D1 expression and phosphorylation in a time dependent manner. Further, treating cells with the aptamer GL21 resulted as well in a stronger and more rapid inhibition of cyclin D1 reaching around 26% at 1 h.

**Figure 5:** Biological activities of selected aptamers. Serum starved U87MG cells were either left untreated or treated with 200 nM of the indicated RNA aptamers or G0 for the indicated incubation times. (*A*) Cell lysates were immunoblotted with anti-phosphocyclin D1 and cyclin D1 antibodies. To confirm equal loading the filters were stripped and reprobed with anti-α-tubulin antibodies. (*B*) Cell lysates were immunoblotted with anti-phosphoERK antibodies and the filters were stripped and re-probed with anti-ERK antibodies. In (*A*) and (*B*), intensity of bands has been calculated using the NIH-Image Program on at least two different exposures to assure the linearity of each acquisition. Four independent experiments were performed. Fold values are expressed relative to the reference points, arbitrarily set to 1 (labeled with asterisk, lane 1). “C” indicates mock-treated cells. Plots of fold values corresponding to the cyclin D1 expression and to ERK activity are reported for each lane of immunoblotting shown in (*A*) and in (*B*), respectively. (*C*) U87MG cells were treated for 24 hs or 48 hs with the indicated aptamers or the G0 starting pool and proliferation was determined by [^3^H]-thymidine incorporation. In (*A*), (*B*) and (*C*), vertical bars indicate the standard deviation values.

As shown in Fig. 5*B* treatment with the same five aptamers caused a similar time dependent inhibition of ERK phosphorylation, inhibition being more rapid with GL35 than GL36, thus according to their respective Kd values (see Table 1), and, as expected, at comparable extents treating with the highly related GL44 and GL43 aptamers. In agreement with its Kd value, the GL44-43 short aptamer, inhibited cyclin D1 expression and ERK phosphorylation at a similar extent of the GL44 aptamer (not shown). To further demonstrate the biological activity of these aptamers we treated growing U87MG cells with either GL44-43 short or the GL21 aptamer and monitored the inhibitory effect on cell proliferation by pulse labeling thymidine incorporation. According with inhibition of ERK activity, treating cells with aptamers for 24 and 48 hs strongly reduces [^3^H]thymidine incorporation (Fig. 5*C*).

Taken together the results indicate that these five aptamers harbor intrinsic biological activity and may act as inhibitory ligands of critical cell surface molecules.

## Discussion

Cancer cell surface epitopes that may discriminate a specific cell phenotype whilst embedded in a heterogeneous cell population are highly promising targets for developing personalized innovative therapeutics. Human gliomas are highly heterogeneous tumors whose sensitivity to therapeutic approaches is hard to predict. Several glioma derived cell lines have been shown to differ in the pattern of expression of receptor tyrosine kinases and in their involvement in cell proliferation [18], thus gliomas may constitute a model of choice in which to demonstrate the possibility to obtain a panel of aptamers that may distinguish a given glioma phenotype.

Here we adopted a differential SELEX protocol to target whole living human glioma derived cells, the U87MG cell line, and we obtained a panel of nuclease-resistant RNA ligands capable of binding at high affinity to the surface of target cells and to distinguish them from other glioma cell lines.

Furthermore, because of the importance of several membrane bound proteins as regulators of cancer cell proliferation we determined in U87MG cells whether any of such aptamers may interfere with the transmission of intracellular signaling and demonstrated that five of these molecules inhibited the activity of critical molecules in cell proliferation, ERK 1/2 and cyclin D1, but not Akt. Lack of inhibition of Akt likely rely on the fact that these cells bear an inactive PTEN, a negative regulator of Akt, and thus the levels of Akt phosphorylation are only poorly regulated by extracellular stimuli [15].

The use of living cells as targets for SELEX has been already described by us and by others [19]. Indeed, we have already demonstrated that it is possible to obtain aptamers for a given transmembrane receptor tyrosine kinase if an appropriate protocol is adopted thus providing the first evidence of the possibility to use SELEX to distinguish between cells that differ for a single (or few) membrane epitope [14], [20].

Here we adopted a similar approach to distinguish between closely related tumor cell lines by targeting unknown epitopes on the cell surface. To surmount the possible drawback of obtaining aptamers targeting few highly represented epitopes we monitored the evolution process by RFLP and stopped the SELEX rounds as soon as the enrichment of the library was visible, i.e. at round 14. This strategy allowed us to obtain aptamers against multiple surface epitopes with Kd values in the nanomolar range, a further increase in affinity is expected by applying further SELEX rounds to each individual aptamers (work in progress). As a first attempt to identify those aptamers that better discriminate the U87MG cells, we screened 21 individual aptamers for their binding at 500 nM to U87MG cells over the naïve G0 random pool. Even if we identified eight aptamers that specifically bind cells at that concentration, given that in this assay we used an unique aptamers concentration we cannot conclude on the specificity of the binding properties of the remaining thirteen aptamers on either U87MG or T98G cells.

Our strategy allowed us to obtain eight, of which six are unrelated, aptamers that bind *bona fide* distinct epitopes present on the cell surface. Further, by this approach we generated a panel of ligands that bind cells used for selection but neither those used for counterselection nor unrelated cancer cells, from neuroblastoma, breast, and lung cancer cell lines. Most importantly, by combining their pattern of binding allows to identify a given glioma cell line among the seven analyzed. Further, the differences in binding are not randomly distributed but in contrast they fit well with important growth properties of each cell line, as tumorigenicity in nude mice, thus suggesting that the extent of binding of an aptamer (see for example GL17) may associate with at least one biological property.

We measured binding efficiency on each cell line using the same concentration of 50 nM for all aptamers. This strategy even if it doesn't exactly reflect the differences in Kd between aptamers (calculated on the U87MG cells) revealed as a simple and direct way to obtain a specific pattern of binding for each cell line. As expected the two cell lines used for selection and counterselection have the best and worst binding for all the aptamers, respectively.

Aptamers have been shown to frequently inhibit the function of their target molecules, presumably by interfering with binding of the cognate ligand [21]. As mentioned above the strategy adopted should allow to enrich for aptamers that target molecules even present at low abundance on the cell surface as for example receptors and other transducing molecules, as already shown for ligands to the receptor tyrosine kinase Ret [14]. The effectiveness of the strategy adopted is well highlighted by the fact that out of eight aptamers that bind to the U87MG, five interfere with the activity of critical molecules for intracellular signaling and cell proliferation likely binding to and/or inhibiting a membrane bound receptor in its active conformation.

In conclusion, we developed a differential SELEX-based procedure that allowed us to generate a highly informative panel of few specific and selective aptamers for malignant glioma cells. The identification of cellular targets for each of these aptamers is in progress. Major advantages of SELEX are the relative rapidity of the entire process and to be only based on artificial molecules. Therefore, the concrete prospective that by such a procedure it is possible to identify and validate important surface target molecules will certainly reveal this as a rather unique tool to discover new molecular targets for antibodies or short peptides.

## Materials and Methods

### Ethics Statement

Primary tumor cultures were derived from surgical biopsies. The study protocol was approved by the local Ethics Committee of the University of Cologne. Written informed consent was acquired prior to surgery from every patient for further studies on primary glioma cultures.

### Cell Culture and Immunoblotting

Human glioma U87MG (American Type Culture Collection, ATCC no. HTB-14), T98G (ATCC no. CRL-1690), A172 (ATCC no. CRL-1620), U251MG (kindly provided by A. Porcellini), TB10 (kindly provided by A. Porcellini), Gli36 [22] cells were grown in Dulbecco's modified Eagle medium (DMEM) supplemented with 2 mM L-glutamine, 10% fetal bovine serum (Invitrogen, Carlsbad, CA). Human glioma, LN-18 (ATCC no. CRL-2610), LN-229 (ATCC no. CRL-2611) were grown in Advanced DMEM supplemented with 2 mM L-glutamine, 10% fetal bovine serum (Invitrogen, Carlsbad, CA). U87MGΔEGFR and Gli36ΔEGFR, expressing a truncated mutant EGFR receptor due to an in-frame deletion of exons 2–7 from the extracellular domain (ΔEGFR) [23], were grown in DMEM supplemented with 2 mM L-glutamine, 10% fetal bovine serum, 500 µg/ml gentamycin (Invitrogen, Carlsbad, CA). Growth conditions for cell lines used were previously reported: human neuroblastoma SH-SY5Y and SK-N-BE cells [24], human breast MCF7 and SKBR3 cells [25], human NSCLC H460 and Calu1 cells [26] and NIH3T3 cells [14].

Primary tumor cultures from surgical biopsies of patients with brain tumors were derived as described previously [27]. Each tumor specimen was cut into small pieces, removing blood vessels, then resuspended in trypsin solution (4% in 0.01 M PBS, pH 7.2). After incubation (37°C, 10 min), DMEM (Life Technologies, Karlsruhe, Germany) supplemented with 20% FBS (Roche Diagnostics, Mannheim, Germany), 100 U/ml penicillin, 100 µg/ml streptomycin (P/S; Life Technologies) and 1% amphotericin (SIGMA, Steinheim, Germany) was added and the cell suspension was centrifuged (210 rcf, 6 min). The pellet was resuspended in DMEM with 20% FBS, 1% P/S and 1% amphotericin and grown at 37°C in a 5% CO_2_/95% air atmosphere. When primary tumor cell cultures formed nearly confluent monolayers, they were frozen and stored in liquid nitrogen for further use.

To assess the functional effects of aptamers, U87MG (300 000 cells per 3.5-cm plate) were serum starved for 2 hs and then treated with the RNA aptamers or the starting RNA G0 pool prior subjected to a short denaturation-renaturation step. Cell extracts preparation and immunoblotting analysis were performed as described [28]. The primary antibodies used were: anti-ERK1 (C-16) (Santa Cruz Biotechnology, Santa Cruz, California, United States) and anti-phospho-44/42 MAP kinase (indicated as anti-pErk), anti-Akt, anti-phospho-Akt (Ser473, indicated as anti-pAkt), anti-PDK1, anti-phospho-PDK1 (Ser241, indicated as anti-pPDK1), anti-phospho-cyclin D1 (Thr286, indicated as anti-pcyclin D1) and anti-cyclin D1 (all from Cell Signaling, Beverly, MA), anti-α-tubulin (DM 1A) (Sigma, St. Louis, MO).

### Whole-Cell SELEX

The SELEX cycle was performed essentially as described [29]. Transcription was performed in the presence of 1 mM 2′-F pyrimidines and a mutant form of T7 RNA polymerase (2.5 u/µl T7 R&DNA polymerase, Epicentre Biotechnologies, Madison, WI.) was used to improve yields. 2'F-Py RNAs were used because of their increased resistance to degradation by seric nucleases. 2'F-Py RNAs (800-300 pmol) were heated at 85°C for 5 min in 1.5 ml of DMEM serum free, snap-cooled on ice for 2 min, and allowed to warm up to 37°C. Before incubation with the cells, 13.5 ml of medium were added to RNA to reach a final volume of 15 ml.

Counterselection against T98G cells. To avoid selecting for aptamers non-specifically recognizing the U87MG cell surface, the pool was first incubated for 30 min (up to round 9) or for 15 min (for the following rounds) at 37°C with 10^7^ T98G cells (150-mm cell plate), and unbound sequences were recovered for the selection phase. This step was meant to select sequences recognizing specifically the U87MG cells.

Selection against U87MG cells. The recovered sequences were incubated with 10^7^ U87MG cells for 30 min at 37°C and recovered after several washings with 5 ml of DMEM serum free by total RNA extraction (Ambion, Austin, TX).

During the selection process, we progressively increased the selective pressure by increasing the number of washings (from one for the first cycle up to five for the last cycles) and by decreasing the incubation time (from 30 to 15 min from round 9). To follow the evolution of the pool we monitored the appearance of four-base restriction sites in the population by RFLP as previously described [30].

### Binding Analysis

Binding of individual aptamers (or the starting pool as a control) to glioma cells was performed in 24-well plates in triplicate with 5′-[^32^P]-labeled RNA. 3.5×10^4^ cells per well were incubated with various concentrations of individual aptamers in 200 µl of DMEM serum free for 20 min at RT in the presence of 100 µg/ml polyinosine as a nonspecific competitor (Sigma, St. Louis, MO). After five washings of 500 µl DMEM, bound sequences were recovered in 300 µl of SDS 1%, and the amount of radioactivity recovered was counted. The background values obtained with the starting pool were subtracted from the values obtained with the specific aptamers. Apparent Kd values for each aptamer were determined by Lineweaver-Burk analysis according to the equation:


### [^3^H]-Thymidine Incorporation Assay

U87MG cells were plated in 24-well dishes (2×10^4^ cells/well) and treated for 24 hs or 48 hs with aptamer (as indicated) or the starting pool (G0) as control. During the final 4 hs, cells were pulsed with 1 µCi/ml [^3^H]-thymidine (45 Ci/mmol) (Amersham-Pharmacia Biosciences) added in complete growth medium and incubated at 37°C. At the end of each pulse, cells were harvested and [^3^H]-thymidine incorporation was analyzed by a Beckman LS 1701 Liquid Scintillation Counter.
